The article "Opioids for treating refractory dyspnea in patients with heart failure: A protocol for systematic review and meta-analysis" was retracted in 2023. Reasons: plagiarism; false authorship; no approval from a third party.

# Opioids for treating refractory dyspnea in patients with heart failure: A protocol for systematic review and meta-analysis

**DOI:** 10.1097/MD.0000000000031699

**Published:** 2022-11-25

**Authors:** Jianguo Lyu, Xianghong Sun, Mingming Chen, Sijia Li

**Affiliations:** a Intensive Care Unit, Shengjing Hospital of China Medical University, Liaoning, China; b Interventional Ward, Shengjing Hospital of China Medical University, Liaoning, China.

**Keywords:** dyspnea, heart failure, meta-analysis, opioid

## Abstract

Dyspnea is a hallmark symptom of heart failure. The existing clinical studies have indicated that opioid can effectively improve the clinical symptoms of heart failure patients with dyspnea. However, there has not been any relevant systematic review and meta-analysis. We performed a protocol for systematic review and meta-analysis to evaluate the safety and efficacy of opioid therapy for heart failure patients with refractory dyspnea.

**Methods:**

We searched 3 foreign electronic databases (Cochrane Library, Embase, Pubmed) and 4 Chinese electronic databases (China National Knowledge Infrastructure, Wang Fang Database, Chinese Biomedical Literature Database and Chinese Scientific Journal Database) to collect potential studies from their inceptions to October 2022. The risk of bias in the included articles was assessed according to the Risk of Bias Assessment Tool in Cochrane Handbook of Systematic Reviews (5th edition). The quality of evidence was assessed by the Grading of Recommendations Assessment, Development and Evaluation approach. Data were analyzed using the RevMan Version 5.4.1.

**Results:**

This study will evaluate whether opioid is effective and safe for treating refractory dyspnea in patients with heart failure.

**Conclusion:**

This meta-analysis will provide comprehensive evidence of opioid therapy for heart failure patients with dyspnea.

## 1. Introduction

Heart failure (HF) is a syndrome characterized by symptoms (such as breathlessness, ankle swelling, and fatigue) and signs (e.g., raised jugular venous pressure, pulmonary crackles, and peripheral edema) caused by structural or functional cardiac abnormalities that lead to elevated intracardiac pressures or a reduced cardiac output at rest or during stress.^[1–3]^ HF is a leading and increasing cause of morbidity and mortality worldwide. The prevalence of HF is age-dependent, ranging from < 2% of people younger than 60 years to more than 10% of those older than 75 years.^[4]^ As a result of aging of the general population and improved treatment of acute cardiovascular events, the prevalence of heart failure is projected to increase by 25% in the next 20 years.^[5]^ For HF patients, healthcare professionals should focus on not only prolonging survival but also improving their quality of life.

Refractory dyspnea (defined as dyspnea that occurs despite optimization of traditional medical management, such as inhaled medications) is a frequently encountered and challenging problem in HF.^[6,7]^ Refractory dyspnea has profound implications on patient quality of life and contributes to significant psychological distress.^[8]^ Although an off-label usage, there is a theoretical role for opioids in the management of refractory dyspnea.^[9,10]^ By binding to opioid receptors that are heavily concentrated in the medulla, where respiratory rhythm is generated, opioids may theoretically lessen refractory dyspnea by decreasing minute ventilation and/or dulling respiratory response to chemoreceptor stimulation from hypoxemia and hypercapnea.^[11]^ Opioid receptors are also located in the deeper cerebral cortex (e.g., insula, thalamus, anterior cingulate cortex, etc.) and opioid action at these sites may help modulate the perception of dyspnea.^[12]^

Currently, the opioid therapy for HF patients with refractory dyspnea have not been widely used. Therefore, we performed a protocol for systematic review and meta-analysis to assess the safety and efficacy of opioid therapy for HF patients with refractory dyspnea.

## 2. Methods

The protocol of this review was registered in PROSPERO (CRD42021252201). Meanwhile, it was reported follow the guidelines of the Preferred Reporting Items for Systematic Reviews and Meta-Analyses.^[13]^ Ethical approval is not required because this review will retrieve publicly available scientific literature.

### 2.1. Inclusion and exclusion criteria

PICOS will be applied, including population, intervention, comparison, outcome, and study.^[14]^

#### 2.1.1. *Type of participants*.

Adults patients (age > 18 years) from HF with dyspnea were included. Regardless of gender, race, occupation, education, nationality, etiology, and severity.

#### 2.1.2. *Type of intervention*.

Patients in intervention group received opioid therapy, regardless of the route of administration used for the treatment of dyspnea.

#### 2.1.3. *Type of comparator (S)/control*.

The control group’s treatment is not limited, including no treatment and placebo.

#### 2.1.4. *Type of outcome measurements*.

Primary outcomes include dyspnea relief at 8, 12, 24 hours/day 1, 48, and 72 hours, and the incidence of worsening renal function (defined as an increase in serum creatinine of ≥ 0.3mg/dl). Secondary outcomes include heart rate, left ventricular ejection fraction, blood urea nitrogen, systolic blood pressure, serum creatinine and adverse events.

#### 2.1.5. *Type of study design*.

Only randomized controlled trials are included. The language will be limited to Chinese and English.

### 2.2. *Search methods for identification of studies*

We searched 3 foreign electronic databases (Cochrane Library, Embase, Pubmed) and 4 Chinese electronic databases [China National Knowledge Infrastructure (CNKI), Wang Fang Database, Chinese Biomedical Literature Database (CBM) and Chinese Scientific Journal Database (VIP)] to collect potential studies from their inceptions to October 2022. The following search terms will be used: heart failure, opioid and dyspnea. A draft search strategy using Pubmed, 1 of the planned electronic databases to be searched, is presented in Table 1.

**Table 1:** Search strategy (PubMed).

Number search terms
#1 opioid[Ti/Ab]
#2 morphine[Ti/Ab]
#3 fentanyl[Ti/Ab]
#4 demerol[Ti/Ab]
#5 codeine[Ti/Ab]
#6 oxycodone[Ti/Ab]
#7 pethidine[Ti/Ab]
#8 remifentanil[Ti/Ab]
#9 sufentanil[Ti/Ab]
#10 buprenorphine[Ti/Ab]
#11 #1 OR #2 OR #3 OR #4 OR #5 OR #6 OR #7 OR #8 OR #9 OR #10
#12 heart failure[Ti/Ab]
#13 cardiac failure[Ti/Ab]
#14 cardiac insufficiency[Ti/Ab]
#15 #12 OR #13 OR #14
#16 dyspnea[Ti/Ab]
#17 breathless[Ti/Ab]
#18 #16 OR #17
#19 #11 AND #15 AND #18

Ab = abstract, Ti = title.

### 2.3. Studies selection

Studies will be identified using Note Express 3.2.0. After the initial removal of duplicate studies, 2 reviewers will independently screen titles and abstracts based on the eligibility criteria. If studies contain insufficient information to make a decision about eligibility, we will try to contact authors of the original reports to obtain further details. During the procedure, disagreements will be resolved by discussion or consensus with the third reviewer. Study selection will be performed in accordance with the Preferred Reporting Items for Systematic Reviews and Meta-Analyses flowchart (Fig. 1).

**Figure 1.** Flow diagram.

### 2.4. Data extraction

Two researchers extracted literature information based on inclusion and exclusion criteria, including the following: Study characteristics: author, year, study design, sample size and follow-up time; Patient characteristics: age, sex, BMI, race, and nationality; Intervention: intervention measures in the experimental group, intervention measures in the control group; Outcome of the study: 2 researchers cross-checked the extraction results of the documents. Disagreements are resolved through discussion among all authors.

### 2.5. Evaluation of risk of bias

The risk of bias in the included articles was assessed according to the Risk of Bias Assessment Tool in Cochrane Handbook of Systematic Reviews (5th edition).^[15]^ Two investigators evaluated the risk of bias for each item as unclear, low risk, and high risk of bias. In case of disagreement, the third investigator was responsible for resolving it.

### 2.6. Evaluation of the evidence quality of the included studies

The quality of evidence was assessed by the Grading of Recommendations Assessment, Development and Evaluation (GRADE) approach.^[16]^ This tool aims to assess the quality of evidence for each outcome indicator in the study. The 2 authors will independently evaluate the evidence of the results and should describe in detail the degradation or upgrade factors that affect the quality of the evidence to ensure the reliability and transparency of the results. Any disagreements will be resolved through discussion by 2 authors. The overall quality of evidence was judged as “high,” “moderate” or “very low.”

### 2.7. Data synthesis and statistical analysis

Meta-analyses were conducted where applicable; otherwise, outcomes were presented in narrative form. Data were analyzed using the RevMan Version 5.4.1. Next, relative risk (RR) for dichotomous outcomes with corresponding 95% confidence intervals (CIs) were computed for individual trials. *χ*2 and Higgins I^2^ tests were used to assess heterogeneity among the included studies. If significant heterogeneity (*P* ≤ .10 for *χ*2 test results or I^2^ ≥ 50%) was obtained, we used a random-effects model, otherwise a fixed-effects model was used. And a *P* < .05 was taken to indicate statistical significance. To assess the robustness of the results, meta-regression analyses (STATA version 12.0) were carried out for sensitivity analysis to test the influence of potential effect modifiers. The *P* value of Egger’s linear regression test was used to assess the presence of publication bias in included articles for each outcome.

## 3. Discussion

The incidence of HF increases year by year with a large aging population in the world. Dyspnea is a hallmark symptom of HF. Therefore, the search for a safe and effective drug has become a much-talked-about and received widespread attention from the global medical community. The existing clinical studies have indicated that opioid can effectively improve the clinical symptoms of patients with HF, such as dyspnea, and has fewer side effects.^[17–19]^ However, the exact mechanism remains to be further explored. There has not been any meta-analysis of the clinical efficacy and safety of opioid for treating refractory dyspnea in patients with HF. We hope that this study can provide more rigorous medical evidence. However, there may be some potential deficiencies in this study. For instance, different doses and courses of treatment in the intervention group in the included trials may lead to relatively significant heterogeneity in the meta-analysis results. Further high quality randomized controlled trials are still required.

## Author contributions

**Data curation:** Xianghong Sun.

**Formal analysis:** Mingming Chen.

**Investigation:** Mingming Chen.

**Writing – original draft:** Jianguo Lyu.

**Writing – review & editing:** Sijia Li.
